# Diagnostic Value of Multislice Spiral Computed Tomography Combined with Serum AFP, TSGF, and GP73 Assay in the Diagnosis of Primary Liver Cancer

**DOI:** 10.1155/2022/6581127

**Published:** 2022-06-07

**Authors:** Chuanwen Yu, Chuang Sun

**Affiliations:** Department of Radiology, The Second Hospital of Dalian Medical University, Dalian 116004, Liaoning, China

## Abstract

**Objective:**

To explore the diagnostic value of multislice spiral computed tomography (MSCT) scan combined with serum alpha-fetoprotein (AFP), tumor-specific growth factor (TSGF), and Golgi protein73 (GP73) assays in the diagnosis of primary liver cancer (PLC).

**Methods:**

Totally, 60 patients with PLC admitted to The Second Hospital of Dalian Medical University from January 2019 to January 2020 were included in group A, 60 patients with liver cirrhosis were included in group B, and 60 healthy subjects were included in group C. The serum AFP, TSGF, and GP73 levels were determined, and all participants received MSCT scanning. The diagnostic efficacy of MSCT, assays of serum AFP, TSGF, and GP73, and their combined detection was analyzed.

**Results:**

Group A had the highest levels of AFP, TSGF, and GP73, followed by group B, and then group C. The sensitivity, specificity, positive predictive value, and negative predictive value of MSCT for PLC were 80.0%,91.7%, 82.8%, and 90.2%, respectively, while those of combined detection of MSCT plus serum AFP, TSGF, and GP73 for PLC were 100.0%, 93.3%, 88.2%, and 100.0%. The combined detection was associated with significantly a higher detection rate of PLC versus stand-alone detection.

**Conclusion:**

MSCT plus serum AFP, TSGF, and GP73 has a higher detection rate versus stand-alone detection, which shows great potential in the diagnosis of PLC.

## 1. Introduction

The incidence of primary liver cancer (PLC) accounts for more than 50% of the total prevalence of liver cancer. The early stage of PLC is mostly asymptomatic, and the disease may have progressed to an advanced stage by the time of diagnosis where surgical outcomes are unfavorable [1, 2]. Thus, early diagnosis is crucial for the improvement of the prognosis of patients [3]. At present, diagnosis of PLC is mostly achieved by imaging examination, and multislice spiral computed tomography (MSCT) can clearly display the liver conditions, which is of high clinical application value [4, 5]. It was found that the detection rate of contrast-enhanced CT scans was about 80.0%, but its diagnostic efficiency might be compromised in the detection of small tumors, which requires additional diagnostic means to enhance the diagnostic accuracy [6, 7]. Tumor markers such as alpha-fetoprotein (AFP), tumor-specific growth factor (TSGF), and Golgi protein 73 (GP73) are commonly used for tumor diagnosis. AFP is commonly used for PLC diagnosis but is associated with poor sensitivity and specificity. Recent research has shown that the combined assay of AFP with other tumor markers might potentiate the diagnostic efficiency [8]. TSGF is a polypeptide secreted during the production and proliferation of malignant tumors, and its secretion mechanism is irrelevant to liver injuries caused by benign liver diseases such as liver cysts and cirrhosis [9]. Therefore, the determination of serum TSGF may facilitate the differentiation between PLC and liver cirrhosis. GP73 is a transmembrane protein of the Golgi apparatus and is rarely detected in the liver cells of healthy people. The elevation of its expression indicates cancerous changes of liver cells [10]. The serum levels of GP73 increase with the severity of liver inflammatory responses, but not significantly. The combination of AFP, TSGF, and GP73 contributes to a higher diagnostic efficiency for PLC [11]. Accordingly, this study was conducted to explore the diagnostic value of MSCT plus serum AFP, TSGF, and GP73 levels in PLC.

## 2. Materials and Methods

### 2.1. General Materials

Totally 60 patients with PLC admitted to The Second Hospital of Dalian Medical University from January 2019 to January 2020 were included in group A, 60 patients with liver cirrhosis were included in group B, and 60 healthy subjects were included in group C. There were no significant differences between the three groups in terms of baseline characteristics (*P* > 0.05), as shown in Table 1.

### 2.2. Inclusion Criteria

The inclusion criteria were as follows: (1) participants and their family members fully understood the research procedures and signed the informed consent. (2) patients of group A were diagnosed with PLC by surgery or biopsy; (3) patients of group B were confirmed with cirrhosis after the examination.

### 2.3. Exclusion Criteria

Exclusion criteria were as follows: (1) patients with mental illness that prevented normal communication; (2) with other organic diseases; (3) who were in pregnancy or lactation.

### 2.4. Methods

This study was approved by the ethics committee of The Second Hospital of Dalian Medical University. All the methods were carried out per the Declaration of Helsinki [12].

1. Detection of serum AFP, TSGF, and GP73 levels: 3 ml of morning fasting venous blood was collected from the patients and centrifuged to obtain the serum. The serum AFP was determined using the electrochemiluminescence method (Cobase 411 electrochemical luminescence device with original auxiliary reagent, Approval No. 3402843 2011), with the range of markers given on the kit as the normal range. The serum TSGF was determined using the colorimetric method (Tai'an City Kangyu Medical Equipment Co. Ltd., Approval No. 2400498). The serum GP73 was determined using the enzyme-linked immunoassay (Beijing Kewei Clinical Diagnostic Reagents Co., Ltd., S20060028). Positive determination of content: serum AFP ≥ 20 ng/mL, TSGF ≥ 70 U/mL, GP73 ≥ 80 ng/mL [13].
2. MSCT scan: patients were required to lie supine, a 64-row helical CT scanner (Philips, drug safety food machinery into the word no. 3303600 2008) was used for scanning. The scanning parameters were pitch of 1.5, scanning thickness of 0.5 cm, transverse reconstruction thickness of 0.2 cm, current of 160 mA, and voltage of 120 kV. A plain CT scan was performed from the diaphragm to the lower margin of the phalangeal joint. After scanning, 100 mL of iohexol contrast agent was injected at a rate of 2.5–3.0 ml/s, followed by scanning 25 s after injection for the arterial phase and 30 s after injection for the venous phase. The examination results were interpreted independently by two radiologists, and consensus was made after discussion with a third radiologist in the event of discrepancies.

### 2.5. Observation Criteria

(1) The levels of AFP, TSGF, and GP73 of the participants were analyzed. (2) The diagnostic efficiency of MSCT was analyzed. (3) The diagnostic efficiency of AFP, TSGF, and GP73 was analyzed. (4) The diagnostic efficiency of combined detection was analyzed.

Diagnostic efficacy includes (1) sensitivity: the ratio of positive cases in group A to the total in that group. (2) Specificity: the ratio of (number of negative cases in group B + number of negative cases in group C) to (total number of cases in group B + total number of cases in group C). (3) Positive predictive value: the ratio of the number of positive cases in group A to (number of positive cases in groups A, B, and C). (4) Negative predictive value: the ratio of (number of negative cases in group B + number of negative cases in group C) to (number of negative cases in groups A, B, and C).

### 2.6. Statistical Analysis

SPSS20.0 was used for data analyses, and GraphPad Prism 7 (GraphPad Software, San Diego, USA) was to plot the graphics. The counting data are analyzed using the chi-square test, and the measurement data are analyzed using the *t*-test. Statistically significant results were defined as *P* < 0.05.

## 3. Results

### 3.1. Analysis of AFP, TSGF, and GP73 Levels

Group A had the highest levels of AFP, TSGF, and GP73, followed by group B, and then group C (*P* < 0.001), as shown in Figures 1 and 2.

### 3.2. Analysis of Diagnostic Efficiency of Multislice Spiral CT Scanning

The sensitivity, specificity, positive predictive value, and negative predictive value of MSCT were 80.0% (48/60), 91.7% (110/120), 82.8% (48/58), and 90.2% (110/122), respectively, as shown in Table 2.

### 3.3. Diagnostic Efficacy of Serum AFP, TSGF, and GP73

The diagnostic efficiency of serum AFP, TSGF, and GP73 is shown in Table 3.

### 3.4. Diagnostic Efficacy of Combined Detection

The sensitivity, specificity, positive predictive value, and negative predictive value of multislice spiral CT combined with serum AFP, TSGF, and GP73 were 100.0%, 93.3%, 88.2%, and 100.0%, respectively. The combined detection was associated with significantly a higher detection rate of PLC versus stand-alone detection (*P* < 0.05), as shown in Table 4.

## 4. Discussion

Imaging examination and tumor marker detection are the main methods for PLC diagnosis, but their detection efficiency for small tumors was unsatisfactory [14].

AFP is a serum glycogen protein and its level reaches a peak in the fetal period and declines after delivery. However, injuries and cancerous changes in liver cells can upregulate the expression of AFP [15]. Therefore, the detection of serum AFP levels may contribute to better PLC diagnostic efficiency [16]. However, recent studies found that AFP lacked sensitivity in the diagnosis of early PLC with a high false-positive rate, which compromised its clinical value [17, 18]. In the present study, the sensitivity and specificity of AFP detection for PLC were 66.7% and 70.0%, respectively, which were consistent with the previous research results [19].

TSGF is a polypeptide and exists in the peripheral blood at the early stage of tumor generation [20]. Accordingly, its expression levels in the serum are associated with tumor development. GP73 is a transmembrane glycoprotein that belongs to bile duct epithelial cells in normal tissues [21]. It participates in the inflammatory responses in the body and exerts a great impact on the protein stability of patients [22]. The results of the present study showed that the level of GP73 in patients with PLC was significantly higher than that in healthy people, and the sensitivity of GP73 for PLC was 83.3%, indicating a positive role of GP73 in PLC diagnosis.

TSGF is present in the serum of patients with early-stage PLC and can discriminate tumor properties. Both GP73 and AFP are sensitive to PLC, so the combined detection efficiency is superior to that of stand-alone detection. The sensitivity, specificity, positive predictive value, and negative predictive value of TSGF, GP73, and AFP were 90.0 (54/60), 80.0 (96/120), 69.2 (54/78), and 94.1 (96/102), respectively, indicating that the combined detection of tumor markers produced a favorable diagnostic yield.

The main blood supply source of healthy liver tissue is the portal vein, while that of PLC patients is the hepatic artery [23]. With blood circulation, the liver cancer lesions of patients gradually disperse, and the diffusion rate of cancer cells rapidly increases through blood metastasis. Multilayer spiral CT scans can clearly visualize the liver lesions of PLC patients [24]. In the present study, contrast-enhanced scanning was performed to compensate for the insufficiency of the original plain scanning, and the sensitivity and specificity of MSCT were 80.0% and 91.7%, respectively, which confirmed the high diagnostic efficiency of MSCT. The sensitivity, specificity, positive predictive value, and negative predictive value of multislice spiral CT combined with serum AFP, TSGF, and GP73 were 100.0%, 93.3%, 88.2%, and 100.0%, respectively. The combined detection was associated with significantly a higher detection rate of PLC versus stand-alone detection (*P* < 0.05), which was in line with the research results of Poynard T [25]. The sensitivity of multislice spiral CT scan combined with serum AFP, TSGF, and GP73 detection was 98.3% (118/120), proving that the combined detection could increase the early detection rate of PLC. However, this study still has the following deficiencies. First, this study is a single-center study without a blind method, which is prone to researcher bias. Secondly, this study is a cross-sectional diagnostic study, and the relationship between the dynamic changes in the above indicators and the severity and prognosis of primary liver cancer remains unclear. Future studies are to include more cases with long-term follow-up of relevant markers to systematically reflect changes in these markers during disease onset and progression and to provide a more accurate basis for prognosis prediction.

## 5. Conclusion

MSCT plus serum AFP, TSGF, and GP73 has a higher detection rate versus stand-alone detection, which shows great potential in the diagnosis of PLC.

## Figures and Tables

**Figure 1:** Analysis of AFP and GP73 levels ($\bar{x}\pm s$, *μ*g/L). The horizontal axis from left to right was AFP and GP73, and the vertical axis referred to the level of serum tumor markers (*μ*g/L); the black area in the figure was group A the dark gray indicated group B and the light gray area was for group C. The level of AFP was (142.56 ± 12.10) *μ*g/L in group A, (105.26 ± 10.23) *μ*g/L in group B, and (3.89 ± 0.56) *μ*g/L in group C; the level of GP73 was (156.89 ± 20.56) *μ*g/L in group A, (131.20 ± 12.48) *μ*g/L in group B, and (16.58 ± 4.26) *μ*g/L in group C; ^*∗∗∗*^*P* < 0.001.

**Figure 2:** Analysis of TSGF level ($\bar{x}\pm s$,U/ml). The horizontal axis from left to right was group A group B and group C, respectively, and the vertical axis indicated TSGF level (U/ml). The level of TSGF was (95.56 ± 6.56) U/ml in group A, (54.11 ± 6.26) U/ml in group B, and (39.89 ± 5.48) U/ml in group C; ^*∗∗∗*^*P* < 0.001.

**Table 1:** Comparison of baseline characteristics.

Group	Group A (*n* = 60)	Group B (*n* = 60)	Group C (*n* = 60)	*P* value
Gender (male/female)	35/25	34/26	33/27	>0.05
Age (year)	53.26 ± 5.11	53.24 ± 5.26	53.20 ± 5.21	
Income (¥)				>0.05
<3000	25	26	27	
≥3000	35	34	33	
Education level				>0.05
High school or below	20	21	19	
College or above	40	39	41	
Drinking	28	27	29	>0.05
BIM over standard	4	5	2	>0.05

**Table 2:** Analysis of diagnostic efficiency of multislice spiral CT scanning.

Multislice CT	Pathologic examination		Total
	Positive	Negative	
Positive	48	10	58
Negative	12	110	122
Total	60	120	180

**Table 3:** Diagnostic efficacy of serum AFP, TSGF, and GP73.

	Sensitivity (%)	Specificity (%)	Positive predictive value (%)	Negative predictive value (%)
AFP	66.7 (40/60)	70.0 (84/120)	52.6 (40/76)	80.8 (84/104)
TSGF	63.3 (38/60)	75.0 (90/120)	55.9 (38/68)	80.4 (90/112)
GP73	83.3 (50/60)	81.7 (98/120)	69.4 (50/72)	90.7 (98/108)

The sensitivity, specificity, positive predictive value and negative predictive value of MSCT combined with serum AFP, TSGF and GP73 were 100.0% (60/60), 93.3% (112/120), 88.2% (60/68) and 100.0% (112/112), respectively.

**Table 4:** Diagnostic efficiency of combined detection of tumor markers.

	Sensitivity (%)	Specificity (%)	Positive predictive value (%)	Negative predictive value (%)
AFP + TSGF	70.0 (42/60)	75.0 (90/120)	58.3 (42/72)	83.3 (90/108)
AFP + GP73	85.0 (51/60)	75.0 (90/120)	63.0 (51/81)	90.9 (90/99)
GP73 + TSGF	83.3 (50/60)	78.3 (94/120)	65.8 (50/76)	90.4 (94/104)
AFP + TSGF + GP73	90.0 (54/60)	80.0 (96/120)	69.2 (54/78)	94.1 (96/102)
AFP + TSGF + GP73 + MSCT	100.0 (60/60)	93.3 (112/120)	88.2 (60/68)	100.0 (112/112)

## Data Availability

All the data generated or analyzed during this study are included in this published article.

## References

[1] Ram A. K., Pottakat B., Vairappan B. (2018). Increased systemic zonula occludens 1 associated with inflammation and independent biomarker in patients with hepatocellular carcinoma. *BMC Cancer*.

[2] Tsuchiya N., Sawada Y., Endo I., Saito K., Uemura Y., Nakatsura T. (2015). Biomarkers for the early diagnosis of hepatocellular carcinoma. *World Journal of Gastroenterology*.

[3] Jeong W. K., Jamshidi N., Felker E. R., Raman S. S., Lu D. S. (2019). Radiomics and radiogenomics of primary liver cancers. *Clinical and Molecular Hepatology*.

[4] Daamen L. A., Groot V. P., Heerkens H. D., Intven M. P. W., van Santvoort H. C., Molenaar I. Q. (2018). Systematic review on the role of serum tumor markers in the detection of recurrent pancreatic cancer. *International Hepato-Pancreato-Biliary Association*.

[5] Sojoodi M., Wei L., Erstad D. J. (2020). Epigallocatechin gallate induces hepatic stellate cell senescence and attenuates development of hepatocellular carcinoma. *Cancer Prevention Research*.

[6] Guo W., Pang Y., Yao L. (2021). Imaging fibroblast activation protein in liver cancer: a single-center post hoc retrospective analysis to compare [68Ga] Ga-FAPI-04 PET/CT versus MRI and [18F]-FDG PET/CT. *European Journal of Nuclear Medicine and Molecular Imaging*.

[7] Millard T., Gupta A., Brenin C., Marshall P., Dillon P. (2019). Radiographically occult carcinomatous spread of breast cancer to the liver: a challenging case. *Case Reports in Oncological Medicine*.

[8] Hirose S., Ishige K., Yamaura M. (2020). A case report: long-term complete response of metastatic hepatocellular carcinoma obtained after discontinuation of 2-month sorafenib monotherapy. *Clin J Gastroenterol*.

[9] Aboushousha T., Mamdouh S., Hamdy H. (2018). Immunohistochemical and biochemical expression patterns of TTF-1, RAGE, GLUT-1 and SOX2 in HCV-associated hepatocellular carcinomas. *Asian Pacific Journal of Cancer Prevention*.

[10] Wakabayashi T., Ouhmich F., Gonzalez-Cabrera C. (2019). Radiomics in hepatocellular carcinoma: a quantitative review. *Hepatol Int*.

[11] Zhang Y., Liu Z., Ji K. (2021). Clinical application value of circulating cell-free DNA in hepatocellular carcinoma. *Frontiers in Molecular Biosciences*.

[12] World Medical Association (2013). World Medical Association Declaration of Helsinki: ethical principles for medical research involving human subjects. *JAMA*.

[13] Zhang X., Chen Z. (2021). Tumor-specificity growth factor combined with tumor markers in nuclear medicine imaging to identify prostate cancer osteonosus. *Journal of Healthcare Engineering*.

[14] El-Sisi A. E., Sokar S. S., Ibrahim H. A., Abu-Risha S. E. (2020). Enhanced anticancer activity of combined treatment of imatinib and dipyridamole in solid Ehrlich carcinoma-bearing mice. *Naunyn-Schmiedeberg’s Archives of Pharmacology*.

[15] Taniai M., Hashimoto E., Tobari M. (2018). Clinicopathological investigation of steatohepatitic hepatocellular carcinoma: a multicenter study using immunohistochemical analysis of adenoma-related markers. *Hepatology Research*.

[16] Kanwal F., Kramer J. R., Mapakshi S. (2018). Risk of hepatocellular cancer in patients with non-alcoholic fatty liver disease. *Gastroenterology*.

[17] Harris P. S., Hansen R. M., Gray M. E., Massoud O. I., McGuire B. M., Shoreibah M. G. (2019). Hepatocellular carcinoma surveillance: an evidence-based approach. *World Journal of Gastroenterology*.

[18] Weaver A. J., Stafford R., Hale J., Denning D., Sanabria J. R., GBD Collaborators (2020). Geographical and temporal variation in the incidence and mortality of hepato-pancreato-biliary primary malignancies:1990-2017. *Journal of Surgical Research*.

[19] Spadaccini M., Lleo A., Ceriani R. (2018). Alpha-fetoprotein screening in patients with hepatitis C-induced cirrhosis who achieved a sustained virologic response in the direct-acting antiviral agents era. *Hepatobiliary and Pancreatic Diseases International*.

[20] Ha E., Kim F., Blanchard J., Juon H. S. (2019). Prevalence of chronic hepatitis B and C infection in Mongolian immigrants in the Washington, District of Columbia, metropolitan area, 2016–2017. *Preventing Chronic Disease*.

[21] Golubnitschaja O., Polivka J., Yeghiazaryan K., Berliner L. (2018). Liquid biopsy and multiparametric analysis in management of liver malignancies: new concepts of the patient stratification and prognostic approach. *The EPMA Journal*.

[22] Duininck G., Lopez-Aguiar A. G., Lee R. M. (2018). Optimizing cancer care for hepatocellular carcinoma at a safety-net hospital: the value of a multidisciplinary disease management team. *Journal of Surgical Oncology*.

[23] Turcanu A., Pitel E., Dumbrava V. T. (2019). Profile of hepatocellular carcinoma in the Republic of Moldova: first-hand information on the presentation, distribution and etiologies. *Romanian Journal of Internal Medicine*.

[24] Drake T. M., Bird T. G. (2019). Editorial: simplifying screening for primary liver cancer - do the LCR1 and LCR2 tests hold the key?. *Alimentary Pharmacology & Therapeutics*.

[25] Yang F., Shi L., Liang T. (2017). Anti-tumor effect of evodiamine by inducing Akt-mediated apoptosis in hepatocellular carcinoma. *Biochemical and Biophysical Research Communications*.

